The article "Mst2 Overexpression Inhibits Thyroid Carcinoma Growth and Metastasis by Disrupting Mitochondrial Fitness and Endoplasmic Reticulum Homeostasis" was retracted in 2023. Reasons: signs of a paper mill; suspected computer-generated content; unreliable results or conclusions; concerns about the data.

# Mst2 Overexpression Inhibits Thyroid Carcinoma Growth and Metastasis by Disrupting Mitochondrial Fitness and Endoplasmic Reticulum Homeostasis

**DOI:** 10.1155/2021/1262291

**Published:** 2021-09-06

**Authors:** Haichao Zhang, Xin Qu, Lu Han, Xu Di

**Affiliations:** Department of Thyroid and Breast Surgery, Tianjin Fourth Central Hospital, The Fourth Central Hospital Affiliated to Nankai University, The Fourth Center Clinical College of Tianjin Medical University, Tianjin 300140, China

## Abstract

Although the incidence of thyroid carcinoma has increased over the past several decades, it has an excellent prognosis and overall 5-year survival, with a stable mortality rate, except in cases with advanced stages or rare malignant tumor types. Biomarkers have emerged as effective targets of molecular therapy against thyroid carcinoma due to their rapid and convenient detection; however, there has been little clinical application. Macrophage stimulating 2 (Mst2) is a proapoptotic protein with implications in carcinogenesis and metastasis. We found that Mst2 overexpression-induced endoplasmic reticulum (ER) stress in MDA-T32 thyroid carcinoma cells, accompanied by elevated caspase-12 activity, increased apoptotic rate, and reduced cell viability. In addition, Mst2 overexpression contributed to mitochondrial damage, as evidenced by increased mitochondrial oxidative stress and activated the mitochondrial apoptotic pathway. Inhibition of the JNK pathway abolished these effects. These results show Mst2 to be a novel tumor suppressor that induces mitochondrial dysfunction and ER stress via the JNK pathway. Thus, Mst2 could potentially serve as a biomarker for developing targeted therapy against thyroid carcinoma.

## 1. Introduction

The incidence of thyroid carcinoma has been increasing worldwide; however, its mortality rate has largely remained stable. Thyroid carcinoma can be categorized into differentiated (papillary and follicular), poorly differentiated, and rarely occurring medullary and anaplastic tumor types. Approximately 80% of the patients are diagnosed with poorly differentiated thyroid carcinoma. Although surgery, chemotherapy, and targeted therapy have proved to be effective in patients with early detection, those with advanced metastatic thyroid carcinoma have few treatment choices and poor prognosis. In addition, despite the initial response to cytotoxic therapy being favorable in 30–40% of patients, a majority of them experience progression during or after treatment. The most common cause of progression to advanced stages is the dysregulation of oncogenes and tumor suppressor genes.

Mitochondria function as a cellular powerhouse to provide a constant supply of ATP for performing numerous biological processes such as metabolism, proliferation, growth, metastasis, differentiation, angiogenesis, and apoptosis [1]. Their involvement in the development and progression of thyroid carcinoma is evident from the fact that mitochondrial proteins serve as potential targets of chemotherapeutic receptor tyrosine kinase inhibitor drugs such as vandetanib and cabozantinib [2, 3]. Moreover, the inhibition of mitochondrial function via disruption of oxidative phosphorylation has been shown to enhance the response to chemotherapy [4]. Endoplasmic reticulum (ER) facilitates the processing of newly formed prosurvival and proproliferation proteins required for tumor growth and metastasis. Impaired ER activity or ER stress has been shown to contribute to thyroid carcinoma metastasis [5, 6]. Another study reported that ER stress reduced the radiosensitivity of thyroid carcinoma cells and inhibited apoptosis [7, 8]. In contrast, a study demonstrated that impaired protein folding and ER activity promoted thyroid carcinoma cell apoptosis [9, 10]. Although the common upstream regulator of mitochondrial fitness and ER integrity has not been elucidated, the above findings show that mitochondrial dysfunction and ER stress are potential therapeutic targets for thyroid cancer.

The article "Mst2 Overexpression Inhibits Thyroid Carcinoma Growth and Metastasis by Disrupting Mitochondrial Fitness and Endoplasmic Reticulum Homeostasis" was retracted in 2023. Reasons: signs of a paper mill; suspected computer-generated content; unreliable results or conclusions; concerns about the data.

Macrophage stimulating 2 (Mst2), also known as mammalian sterile 20 kinase 2, is a serine protease that regulates posttranscriptional phosphorylation of several proteins. For example, Mst2 strengthens the immune system by promoting the activation of the IL-2/Stat5 signaling pathway [11, 12]. Mst2 controls the activity of the Akt prosurvival pathway, a downstream event in Mst2 upregulation [13, 14]. In addition, Mst2 is known to control the differentiation of the epididymal initial segment via the MEK–ERK pathway [15]. Recent studies have implicated Mst2 in regulating mitochondrial ROS production, suggesting a link between Mst2 and mitochondrial dysfunction [16]. In addition, upregulated levels of ER stress markers, such as CHOP, caspase-9, and GRP94, following Mst2 activation in a rat model of diabetic cardiomyopathy [17] highlight its function in maintaining ER homeostasis. Based on these findings, we speculate Mst2 as a common upstream mediator of mitochondrial function and ER stabilization.

## 2. Materials and Methods

### 2.1. Cell Culture and Treatment

Human thyroid carcinoma MDA-T32 (ATCC® CRL-3351™) cells were maintained in Dulbecco's modified Eagle's medium (DMEM) supplemented with 10% fetal bovine serum (FBS) and 1% antibiotics in 5% CO_2_ at 37°C [18]. To overexpress Mst2, MDA-T32 cells were transfected with adenovirus-expressing Mst2 constructs [19].

The article "Mst2 Overexpression Inhibits Thyroid Carcinoma Growth and Metastasis by Disrupting Mitochondrial Fitness and Endoplasmic Reticulum Homeostasis" was retracted in 2023. Reasons: signs of a paper mill; suspected computer-generated content; unreliable results or conclusions; concerns about the data.

### 2.2. Cell Proliferation Assay

A CCK8 assay was conducted following the manufacturer's instructions (DH343-2, Beijing Dongsheng Biotechnology, China). Briefly, cells with or without Mst2 overexpression were seeded in 96-well plates (2,000 cells/well) and cultured for 5 days [20]. Next, 10 *μ*L of CCK8 (5 mg/mL) was added to the culture medium, and cells were further cultured for 2 h. Finally, the OD was measured at 490 nm (BioTek ELx800, USA) [21].

### 2.3. Western Blotting

The total protein was extracted from the cells following the standard protocol (Beyotime Biotechnology Co., Ltd.), and the protein concentration was determined using a bicinchoninic acid (BCA) protein assay kit. The total protein (40 *μ*g) was subjected to 15% SDS-PAGE, and the separated proteins were transferred to nitrocellulose membranes [22]. After blocking in fresh 5% nonfat milk at room temperature for 2 h, membranes were incubated overnight at 4°C with the primary antibodies, followed by incubation with the secondary antibody at room temperature for 2 h. An enhanced chemiluminescence (ECL) kit (Thermo Fisher Scientific, Inc.) was used to visualize the signals [23]. The antibodies (Affinity Biosciences Ltd.) used included anti-SIRT1 (FD6033; 1 : 1000), anti-p-AMPK (AF3423; 1 : 1000), anti-AMPK (AF6423; 1 : 1000), anti-Cox-2 (AF7003; 1 : 1000), anti-iNOS (AF0199; 1 : 1000), anti-Bcl-2 (AF6139; 1 : 1000), anti-Bax (AF0120; 1 : 1000), anticleaved caspase-3 (AF7022; 1 : 1000), anticleaved caspase-9 (AF5240; 1 : 1000), anti-GAPDH (AF7021; 1 : 5000), and goat anti-rabbit IgG (S0001; 1 : 5000). The protein expression was semiquantified using ImagePro Plus software, version 6.0 (Roper Technologies, Inc.) [24].

### 2.4. MTT Assay

A suspension of ∼5,000 MDA-T32 cells was seeded in 96-well plates. MTT (Sigma) was added to the wells, and cells were incubated for 4 h in 5% CO_2_ at 37°C [25]. Next, 150 *μ*L of dimethyl sulfoxide (DMSO) was added to each well for 10 min, and the absorbance of formazan was measured at 490 nm from 0 to 72 h [26].

### 2.5. Reverse Transcription-Quantitative PCR

The total RNA was extracted from cells using the TRIzol reagent (Invitrogen). We used 1 *μ*g of total RNA to generate cDNAs using the PrimeScript RT reagent kit (Takara) [27]. Reverse transcription-quantitative polymerase chain reaction (RT-qPCR) was performed using the SYBR Green I Master Mix kit. The relative gene expression was calculated using the 2^−ΔΔCt^ method [28].

### 2.6. Immunofluorescence Assay

Cells were cultured on glass coverslips and transfected with Mst2-overexpressing adenovirus constructs. Afterward, cells were washed twice with phosphate-buffered saline (PBS), fixed in 4% formaldehyde for 10 min, and quenched with 50 mM NH_4_Cl in PBS for 10 min [29]. After three washes with PBS, cells were permeabilized with 0.1% Triton X-100 in PBS for 5 min at 4°C. The excess binding sites were blocked with SuperBlock Blocking Buffer in PBS (Thermo Fisher Scientific, #37517) for 1 h at room temperature. The cells were incubated with primary antibodies overnight at 4°C, followed by incubation with secondary antibody for 1 h at room temperature [30]. Cells were washed thrice with PBS containing 1% BSA, and coverslips were mounted onto glass slides using Vectashield containing DAPI (Vector Laboratories, Burlingame, CA, USA). Images were captured using the Zeiss Axio Imager M1 automated microscope (Zeiss, Oberkochen, Germany) [31].

The article "Mst2 Overexpression Inhibits Thyroid Carcinoma Growth and Metastasis by Disrupting Mitochondrial Fitness and Endoplasmic Reticulum Homeostasis" was retracted in 2023. Reasons: signs of a paper mill; suspected computer-generated content; unreliable results or conclusions; concerns about the data.

### 2.7. Propidium Iodide Staining

MDA-T32 cells were incubated in a medium containing a 1 : 500 dilution of PI (Thermo Fisher Scientific) at 37°C [32]. After 30 min, PI was removed, and the cells were washed twice with the medium [33]. The number of PI-positive cells was determined using fluorescence microscopy with an excitation of 535 nm and emission of 617 nm at 200x magnification [34].

### 2.8. ATP Assay and Mitochondrial ROS Production

Cellular ATP levels were measured using a commercial kit (Abcam) [35]. Mitochondrial ROS production was measured using the MitoSOX red mitochondrial superoxide indicator (Molecular Probes, USA) [36].

### 2.9. Cell Transfection

Adenovirus constructs overexpressing human Mst2 (Ad-Mst2) used for cell transfection (Vigene Biosciences Co., Ltd., Shandong, China) [37]. In brief, MDA-T32 cells were transfected with Ad-Mst2 and control adenovirus (ad-Cont) at a multiplicity of infection (MOI) of 100 for 8 h in a serum-free medium [38]. Next, the medium was discarded, and cells were grown in a complete medium for 48 h. Mst2-expressing cells were selected using puromycin (5 *μ*g/mL). The Mst2 expression was verified by qPCR and Western blotting [39].

### 2.10. Statistical Analysis

All data are presented as mean ± standard error of the mean (SEM). Differences between the groups were analyzed using Student's *t*-tests or one-way analysis of variance (ANOVA). *P* < 0.05 was considered significant [40]. All experiments were conducted at least in triplicate.

## 3. Results

### 3.1. Mst2 Overexpression Induces ER Stress

We first overexpressed Mst2 in MDA-T32 cells to study its effect on ER homeostasis. As shown in Figures 1(a)–1(c), compared with the control group, Mst2 overexpression upregulated the transcription of CHOP, GRP78, and PERK, the markers of ER stress. In addition, we found elevated expression of CHOP, GRP78, and PERK proteins (Figures 1(d)–1(f)), suggesting that ER stress is induced by Mst2 overexpression. Irreversible ER damage activates caspase-12—an essential step in the cell apoptosis pathway. The enzyme-linked immunosorbent assay (ELISA) demonstrated that Mst2 overexpression enhanced the activity of caspase-12 in MDA-T32 cells (Figure 1(g)) when compared with the control group. Altogether, our results illustrate that Mst2 overexpression is associated with ER stress.

The article "Mst2 Overexpression Inhibits Thyroid Carcinoma Growth and Metastasis by Disrupting Mitochondrial Fitness and Endoplasmic Reticulum Homeostasis" was retracted in 2023. Reasons: signs of a paper mill; suspected computer-generated content; unreliable results or conclusions; concerns about the data.

### 3.2. Mst2 Overexpression Promotes Mitochondrial Damage

We next studied the effects of Mst2 overexpression on mitochondrial function and structure. As shown in Figures 2(a) and 2(b), the immunofluorescence assay revealed the reduced number of mitochondria in Mst2-overexpressing MDA-T32 cells compared with the control group, suggesting that Mst2 overexpression decreased the mitochondrial mass. In addition, MitoSOX red staining revealed elevated mitochondrial ROS production in MDA-T32 cells (Figures 2(c) and 2(d)), accompanied by reduced levels of glutathione (GSH) and decreased activity of superoxide dismutase (SOD) and glutathione peroxidase (GPX) (Figures 2(e)–2(g)). This finding confirmed that oxidative stress was triggered by Mst2 overexpression in MDA-T32 cells. Next, we found that the mitochondria-related apoptotic pathway was activated, as evident by increased activities of Bax and caspase-9 (Figures 2(h) and 2(i)), when compared with the control group. Altogether, our results demonstrate that mitochondrial function is hindered by Mst2 overexpression in MDA-T32 cells.

### 3.3. Mst2 Inhibits the Viability of Thyroid Carcinoma Cells

Impaired mitochondrial function and ER stress ultimately activate tumor cell death [41]. Therefore, we next studied whether Mst2-induced mitochondrial damage and ER stress were associated with increased MDA-T32 cell apoptosis. First, we determined the cell viability using the MTT assay. As shown in Figure 3(a), MDA-T32 cell viability was highly reduced. Moreover, the lactate dehydrogenase (LDH) release assay revealed elevated LDH content in the medium, suggesting increased cell membrane disintegration in Mst2-overexpressing MDA-T32 cells (Figure 3(b)). Because mitochondrial damage and ER stress-induced cell death is primarily executed by apoptosis, we further analyzed the number of apoptotic cells. Thus, propidium iodide (PI) staining was performed. As shown in Figures 3(c) and 3(d), ∼40% of Mst2-overexpressing MDA-T32 cells were apoptotic compared with only ∼6% PI-positive cells in the control group. Overall, our results confirm that Mst2 overexpression activates apoptosis by impairing mitochondrial function and inducing ER stress.

### 3.4. Thyroid Carcinoma Proliferation Is Impaired by Mst2 Overexpression

Rapid proliferation rate is one of the hallmarks of malignant cancer cells [42, 43]. Therefore, we wanted to understand whether tumor proliferation of thyroid carcinoma cells was controlled by Mst2. The CCK8 assay demonstrated highly reduced growth rate of MDA-T32 cells following Mst2 overexpression (Figure 4(a)). At the molecular level, cyclin-related proteins have been reported to participate in cancer proliferation. Western blotting showed that the protein expression of cyclin D and cyclin E1 was markedly reduced by Mst2 overexpression when compared with the control group (Figures 4(b) and 4(c)). Altogether, these results confirm our hypothesis that thyroid carcinoma proliferation was inhibited by Mst2 overexpression.

The article "Mst2 Overexpression Inhibits Thyroid Carcinoma Growth and Metastasis by Disrupting Mitochondrial Fitness and Endoplasmic Reticulum Homeostasis" was retracted in 2023. Reasons: signs of a paper mill; suspected computer-generated content; unreliable results or conclusions; concerns about the data.

### 3.5. Mst2 Impairs Mitochondrial and ER Functions through the JNK Pathway

The above results showed that Mst2 overexpression suppressed mitochondrial and ER functions and thus promoted MDA-T32 cell apoptosis and proliferation arrest. Recent studies have revealed an intricate link between Mst2 overexpression and JNK activation. In addition, the JNK pathway has been reported to function upstream of mitochondrial damage and ER stress pathways. Therefore, we investigated the involvement of JNK in Mst2-induced mitochondrial and ER damage. Treatment of Mst2-overexpressing MDA-T32 cells with SP600125, a JNK inhibitor, reversed the reduction in mitochondrial number as compared with the control group (Figures 5(a) and 5(b)). Furthermore, Mst2-induced mitochondrial ROS production was attenuated by SP600125 (Figures 5(c) and 5(d)), suggesting that Mst2-induced oxidative stress was dependent on the JNK pathway. Similarly, SP600125 treatment reduced Mst2 overexpression-induced transcription of CHOP, GRP78, and PERK (Figures 5(e)–5(g)). Altogether, our results demonstrate that Mst2 disrupts mitochondrial function and induces ER stress in MDA-T32 cells through the JNK pathway.

## 4. Discussion

Thyroid carcinoma is one of the most common endocrine cancers with a high cure rate. Several factors contribute to thyroid carcinoma, including genetic, environmental, and lifestyle-related. Recent advances in medical imaging have led to early diagnosis and treatment of thyroid carcinoma [44]. The standard treatment includes surgery and radioactive iodine therapy; targeted therapies using specific biomarkers [45], such as tyrosine kinase inhibitors, have been recently introduced and appear to be promising due to their rapid and convenient detection. However, their clinical application is less, indicating the need to explore new effective biomarkers to improve the diagnostic efficiency, prognosis, and treatment outcomes. We showed that Mst2 overexpression in thyroid carcinoma cells induced mitochondrial damage and ER stress resulting in apoptosis and cell proliferation arrest [46]. Therefore, therapeutic approaches targeting Mst2 activity can further enhance the response of thyroid carcinoma to chemotherapy and radiotherapy.

The article "Mst2 Overexpression Inhibits Thyroid Carcinoma Growth and Metastasis by Disrupting Mitochondrial Fitness and Endoplasmic Reticulum Homeostasis" was retracted in 2023. Reasons: signs of a paper mill; suspected computer-generated content; unreliable results or conclusions; concerns about the data.

The Mst family includes Mst1 and Mst2, and anticancer effects of Mst activation have been reported by several studies. For example, Mst1 activation induced oxidative stress and suppressed pancreatic cancer progression by promoting pyroptosis [47, 48]. Similarly, reduced serum levels of Mst1 and Mst2 have been correlated with the development of liver cancer due to the increased proliferation of tumor cells [49, 50]. Moreover, overexpressed Mst1 reduced the invasiveness and proliferation of lung cancer cells [51, 52]. In breast cancer, reduced expression of Mst1 is associated with increased tumor proliferation and migration [53]. Mst1 and Mst2 are known to suppress colonic tumorigenesis and tumor stem cell proliferation by inhibiting Yes-associated protein (Yap) [54, 55]. Similar to these findings, we found that Mst2 overexpression suppressed the development of thyroid carcinoma by promoting cancer apoptosis and inhibiting cell proliferation.

Numerous studies have investigated the function of Mst family proteins in regulating mitochondrial function in cancer survival and metastasis [56–58]. For example, the overexpression of Mst1 suppressed gastric cancer cell viability by inactivating the AMPK–Sirt3 pathway and inducing mitochondrial division [59]. Similarly, overexpressed Mst1 caused mitochondria-dependent breast cancer cell apoptosis via the JNK–Drp1 pathway [60]. Another study reported the tumor-suppressive effects of Mst1 on cancer cell proliferation and metastasis by activating the *β*-catenin/Drp1 axis [61]. Furthermore, Mst1 overexpression impaired the proliferation and migration of colorectal cancer cells by activating the JNK/*p*53/Bnip3 pathway [62]. The overexpression of Mst1 hindered ATP production and redox biology in nonsmall cell lung cancer through the ROCK1/F-actin pathway [63]. Furthermore, Mst2 is a potential target of several anticancer drugs such as gemcitabine [64], tanshinone IIA [65], and matrine [66]. In addition to mitochondria, we reported that ER damage, such as ER stress and ER-related apoptosis, was induced by Mst2. Thus, new therapeutic approaches are being explored to simultaneously affect mitochondrial function and ER homeostasis [67].

Our study had certain limitations. First, because Mst2 is an intracellular protein, there is a need to design new drugs to specifically target its expression. Second, animal studies and clinical trials are warranted to study the molecular basis of Mst2 effects on mitochondrial and ER functions in cancer cells. Third, negative effects of Mst2 overexpression on normal tissues should be considered while designing targeted cancer therapies.

The article "Mst2 Overexpression Inhibits Thyroid Carcinoma Growth and Metastasis by Disrupting Mitochondrial Fitness and Endoplasmic Reticulum Homeostasis" was retracted in 2023. Reasons: signs of a paper mill; suspected computer-generated content; unreliable results or conclusions; concerns about the data.

## Figures and Tables

**Figure 1:** Mst2 overexpression induces ER stress. (a)–(c) MDA-T32 cells transfected with Mst2 adenovirus (Ad-Mst2) constructs. Next, a qPCR assay was used to analyze the transcription of CHOP, GRP78, and PERK. (d)–(f) Western blots showing the expression of CHOP, PERK, and GRP78. (g) ELISA performed to analyze the activity of caspase-12. ^*∗*^*P* < 0.05.

**Figure 2:** Mst2 overexpression promotes mitochondrial damage. (a)-(b) An immunofluorescence assay used to analyze the mitochondrial number. (c)-(d) MitoSOX red staining used to study the mitochondrial ROS production in response to Ad-Mst2 transfection. (e)–(g) ELISA performed to analyze the activity of antioxidative enzymes such as GSH, SOD, and GPX. (h)-(i) ELISA performed to detect the alterations in Bax and caspase-9 activities. ^*∗*^*P* < 0.05.

**Figure 3:** Mst2 inhibits the viability of thyroid carcinoma cells. (a) Cell viability measured using the MTT assay. (b) LDH release assay performed to detect cell death. (c)-(d) PI staining used to quantify the number of apoptotic cells. ^*∗*^*P* < 0.05.

**Figure 4:** Thyroid carcinoma proliferation is impaired by Mst2. (a) Cell proliferation measured using the CCK8 assay. (b)-(c) qPCR assay used to analyze the transcription of cyclin D and cyclin E1. ^*∗*^*P* < 0.05.

**Figure 5:** Mst2 impairs mitochondrial and ER functions through the JNK pathway. (a)-(b) Mst2-overexpressing MDA-T32 cells treated with SP600525, a JNK inhibitor. An immunofluorescence assay was used to analyze the mitochondrial number. (c)-(d) MitoSOX red staining used to study the mitochondrial ROS production in response to Ad-Mst2 transfection. (e)–(g) qPCR assay performed to analyze the transcription of CHOP, GRP78, and PERK. ^*∗*^*P* < 0.05.

## Data Availability

The data used to support the findings of this study are available from the corresponding author upon request.
